The article "Screening of Adverse Prognostic Factors and Construction of Prognostic Index in Previously Untreated Concurrent Follicular Lymphoma and Diffuse Large B-Cell Lymphoma" was retracted in 2023. Reasons: signs of a paper mill; compromised peer review; unreliable results or conclusions.

# Screening of Adverse Prognostic Factors and Construction of Prognostic Index in Previously Untreated Concurrent Follicular Lymphoma and Diffuse Large B-Cell Lymphoma

**DOI:** 10.1155/2022/4379556

**Published:** 2022-05-24

**Authors:** Zhenjie Qu, Tingting Zhang, Fenghua Gao, Wenchen Gong, Yaoli Cui, Lihua Qiu, Zhengzi Qian, Shiyong Zhou, Bin Meng, Xiubao Ren, Lanfang Li, Xianhuo Wang, Huilai Zhang

**Affiliations:** ^1^Department of Lymphoma, Tianjin Medical University Cancer Institute and Hospital, National Clinical Research Center for Cancer, Key Laboratory of Cancer Prevention and Therapy, Tianjin's Clinical Research Center for Cancer, Sino-US Center for Lymphoma and Leukemia Research, Tianjin, China; ^2^Department of Pathology, Tianjin Medical University Cancer Institute and Hospital, Tianjin, China; ^3^Department of Immunology/Biotherapy, Tianjin Medical University Cancer Institute and Hospital, Tianjin, China

## Abstract

**Objective:**

Concurrent follicular lymphoma (FL) and diffuse large B-cell lymphoma (DLBCL) (defined as FL/DLBCL) have been considered an important pathological feature in cell lymphoma. However, clinicopathological information and prognostic factors in these cases are scarce. The aim of this study was to construct a prediction index to compare with traditional prognostic models.

**Methods:**

Retrospectively enrolled, previously untreated FL/DLBCL (*n* = 121) patients, as well as those with pure FL 1–3a (*n* = 471), were assessed. De novo DLBCL (*n* = 529) were used as controls. Kaplan–Meier curves were plotted to compare the outcomes among the three groups. Multivariate analysis identified risk factors associated with overall survival (OS) in FL/DLBCL patients. A clinicopathological prognosis index (CPPI) was developed to predict OS based on the Cox proportional hazards model.

**Results:**

The outcomes of FL/DLBCL patients were intermediate between pure FL 1–3a and *de novo* DLBCL patients, with a 5-year PFS of 70%, 59%, and 48% (*P* < 0.05) and 5-year OS of 80%, 70% and 60% (*P* < 0.05), respectively. Cox regression analysis showed that the prognostic factors of OS for FL/DLBCL patients included FL grade, cell of origin, and Ann Arbor stage. A nomogram and clinicopathological prognostic index (CPPI) were developed to predict the OS for FL/DLBCL patients based on these factors. The area under the curve (AUC) of the CPPI for 3- and 5-year OS prediction was 0.782 and 0.860, respectively. This was superior to that of the International Prognostic Index (IPI), Follicular Lymphoma International Prognostic Index (FLIPI), and FLIPI2 in the 0.540–0.819 (*P* < 0.01) range.

**Conclusions:**

A valid OS estimation in FL/DLBCL patients, using the recommended CPPI, may be useful in routine clinical practice.

## 1. Introduction

Follicular lymphoma (FL) is a common non-Hodgkin lymphoma (NHL) subtype, contributing to more than one-fifth of NHL cases in Western nations [1, 2]. It is a diverse category of cancer that arises from germinal center B cells' centrocytes and centroblasts [3]. Although initially indolent and often observed without treatment at diagnosis, this disease remains largely incurable. Furthermore, it is often followed by repeated relapses and/or transformation to high-grade NHL [4]. FL demonstrates a 3–5 percent risk of developing diffuse large B-cell lymphoma (DLBCL) [5–7]. However, most of the concurrent FL and DLBCL cases exhibit a composite histology. No consensus has been established on whether these represent the co-evolvement of independent FL and DLBCL clones or early transformation of previously undiagnosed FL [6]. Histological confirmation of FL with concurrent DLBCL is considered an invasive lymphoma and implies a very adverse prognosis with a 14–27-month median survival interval [8, 9]. Several published studies clarified clinical biomarkers and predictors of overall survival (OS) of histological transition (HT) [10, 11]. Mutations in the CDKN2A/B and TP53 genes, together with MYC and BCL6 rearrangements, have also been linked to HT [12–15]. Factors linked to poor HT OS include higher age, worse performance status, higher serum levels of *β*2-microglobulin, and high-risk Follicular Lymphoma International Prognostic Index (FLIPI) [16, 17].

Lymph node biopsies typically display concurrent FL and diffuse large B-cell lymphoma (FL/DLBCL) histology. In any case, management of FL/DLBCL is based on aggressive histology (DLBCL) with rituximab combination regimens. However, FL/DLBCL has not only been routinely excluded from phase 3 clinical trials, but data published on diagnosis, prognostic factors, and outcomes are conflicting [4, 6, 18]. A previous study suggests that the PFS and OS were between those for FL and DLBCL (5-year OS rates: 85%, 73%, and 63%, respectively) [19]. However, other studies suggest that the FL/DLBCL and germinal center B-cell-like- (GCB-) subtype DLBCL exhibit similar prognoses [6, 20]. One recent report found FL/DLBCL to exhibit 5-year OS and PFS rates of 92.9% and 68.2%, respectively [5]. Relative to *de novo* DLBCL patients, OS was comparable in those with FL/DLBCL (*P* = 0.15), whereas PFS was significantly worse (*P* = 0.030). Further *de novo* DLBCL patient stratification based on cell of origin (COO) revealed FL/DLBCL to exhibit a prognosis comparable to that of individuals with non-GCB-type DLBCL but worse than that of patients with GCB-type DLBCL (*P* = 0.0024).

Several predictive models such as the FLIPI [21], the FLIPI2 [22], and the International Prognostic Index (IPI) [23] have been employed for stratifying the risk categories within FL and DLBCL patients [24]. However, IPI development preceded that of rituximab, and a combination of rituximab and conventional CHOP (cyclophosphamide, doxorubicin, vincristine, and prednisolone) or CHOP-like regimens for DLBCL markedly improved survival outcomes since the 1990s in a wide range of risk groups [25, 26]. Furthermore, the predictive value of the IPI has fallen in risk stratification, particularly in the higher-risk patients [27].

To forecast the outcome of *de novo* FL 1–3a patients, many prognostic models, such as FLIPI and FLIPI2, are available. The FLIPI was developed in retrospective research to predict OS, while the FLIPI2 was developed to predict PFS as the primary effectiveness objective for model development [28, 29]. Overall, the IPI, FLIPI, and FLIPI2 have been the foundation for initial risk assessment in DLBCL and FL 1–3a patients for decades, laying the path for therapy selection, balancing within clinical trials, and comparison between studies.

In recent years, attempts to identify the mechanistic foundation for prognosis in malignant lymphoma via immunohistochemical or molecular approaches uncovered several gene signatures and biomarkers of prognostic significance. These new prognostic indicators, such as FL Evaluation Index (FLEX) [29], m7-FLIPI [30], and the 23-gene signature [31], are mostly independent of the clinically based prognostic system. Therefore, they do not add much to the predictive ability. This is primarily because of technical or repeatability issues that limit the application of these markers. Nevertheless, FL/DLBCL patients were always excluded by the trial. Therefore, some new prognostic indices based on the common clinicopathological databases are urgently needed to recognize different risk groups in patients with FL/DLBCL.

Thus, in our retrospective study, we compared the outcome of FL/DLBCL patients with that of newly diagnosed patients with pure FL 1–3a and *de novo* DLBCL during the same period. Also, we analyzed the clinicopathological characteristics and outcomes of FL/DLBCL and investigated their prognostic value. As a result, a concise clinicopathological prognostic index (CPPI) for OS was developed to help clinicians better manage this important disease and compare its predictive capacity to IPI, FLIPI, and FLIPI2.

## 2. Patients and Methods

### 2.1. Patients

In our study, patients who were consecutively diagnosed with FL/DLBCL (121 cases), pure FL 1–3a (471 cases), or *de novo* DLBCL (529 cases) between January 2010 and August 2019 at Tianjin Medical University Cancer Institute and Hospital (TMUCIH) were retrospectively analyzed. The diagnoses were assigned based on morphological and immunohistochemical findings reviewed by expert hematopathologists in our institute. The baseline characteristics are presented in Supplementary Tables 1, 2, and 3. All patients received chemotherapy (R-chemotherapy or chemotherapy). In the FL/DLBCL group, 71 (59%) cases were treated with R-chemotherapy regimens (i.e., R-CHOP or R-CHOP like), and 50 (41%) cases were treated with chemotherapy regimens (i.e., CHOP, GEMOX, and CVP). The median follow-up duration for FL/DLBCL was 52.0 months. All patients supplied informed permission in agreement with the Helsinki Declaration. This research was conducted with the approval of the TMUCIH's Ethics Committee.

### 2.2. Demographical and Clinicopathological Information

Relevant demographic and clinicopathological data were gathered for analysis. Demographic data included age and gender. Available clinicopathological characteristics of each patient were recorded and evaluated among the three groups (pure FL 1–3a, FL/DLBCL, and *de novo* DLBCL). These included the existence of B-symptoms (night sweats, fever, and weight loss), performance status agreeing with the Eastern Cooperative Oncology Group (ECOG) scale, tumor extension data, nodal and extranodal involvement, number of extranodal sites involved, bone marrow involvement, spleen involvement, and Ann Arbor stage. Hematological factors included hemoglobin, *β*2-microglobulin (*β*2m) levels, and serum lactate dehydrogenase (LDH); histopathological data included the proportion of DLBCL component, FL grade, and DLBCL subtype (GCB, non-GCB) by Han's algorithm. Furthermore, the FLIPI, the FLIPI2, and the IPI were included in the analysis. While immunohistochemical staining was performed, insufficient Ki-67 tissue expression data were available for analysis. OS is the primary outcome of interest in this study. OS was computed from the time of diagnosis to the time of death from any cause or censored for survivors at the final follow-up date.

### 2.3. Definition of FL/DLBCL and Exclusion Criteria

FL/DLBCL was diagnosed based on morphological and immunohistochemical findings reviewed by our expert hematopathologists. Following the descriptions of previous studies [32], FL/DLBCL was defined by lymph node biopsy samples simultaneously exhibiting either “concurrent” or “discordant” FL and DLBCL aspects at time of diagnosis. Concurrent aspects are those for which a single tissue sample exhibited both lymphoma types. Meanwhile, discordant aspects are those for which components are present across different regions [19]. WHO criteria were employed to grade the FL component. Grade 1 FL exhibited 0–5 centroblasts/HPF (follicular small cleaved). Grade 2 FL exhibited 6–15 centroblasts/HPF (follicular mixed). Grade 3 FL exhibited more than 15 centroblasts/HPF (follicular big cleaved) (follicular large cell). Grade 3 is further split into grade 3a FL, which contains centrocytes, and grade 3b FL, which contains sheets of centroblasts. A cluster of big cells in sheets with no follicular architecture characterizes the DLBCL component, as shown by follicular dendritic cell staining. Based on the relative percentage of DLBCL to the whole assessed specimen, the proportion of DLBCL was calculated. According to the Hans algorithm, DLBCL cells were classified into two types: GCB and non-GCB (immunohistochemical staining for CD10, BCL6, and MUM1). Those unclassified were excluded based on histopathology.

All patients did not receive the evaluation, treatment or intervention specified in the study. Patients with FL diagnosed within 6 months and no prior lymphoma history were eligible for enrollment [10]. Individuals were excluded if they exhibited DLBCL coexistent with others who were considered to have acquired transformation from FL or whose DLBCL was coexistent with other indolent aspects (such as CLL/SLL, MZL, or MALT lymphoma) [33]. Individuals presenting a previously known history of FL received “Wait and Watch” regimens, primary CNS lymphoma, secondary histologic transformation, or primary mediastinal large B-cell lymphoma were excluded based on clinical history [6].

### 2.4. Prognostic Index Construction and Internal Validation

The major goal of this study was to create a prognostic index for FL/DLBCL based on shared clinicopathological features and compare it to conventional prognostic models. We selected common clinicopathological characteristics that are shown to be related to OS and integrated them into the nomogram. We calculated the sum points for each patient and then divided these 121 FL/DLBCL patients by a quartile into four risk groups, according to each patient's total points. Low, low-intermediate, high-intermediate, and high-risk groups identified the patients with the top 25%, 26–50%, 51–75%, and the bottom 25% of the total points, respectively. The risk stratification ability of CPPI, IPI, FLIPI, and FLIPI2 in the primary cohort was ascertained through plotting Kaplan–Meier survival curves.

All 121 FL/DLBCL patients were divided at random into a pair of groups in a ratio of 6 : 4 as internal validation cohorts (internal validation cohort A: *n* = 72 (60%), internal validation cohort B: *n* = 49 (40%)). These were compared with traditional prognostic models (IPI, FLIPI, and FLIPI2) using Kaplan–Meier survival curves. The predictive accuracy of the CPPI, IPI, FLIPI, and FLIPI2 was verified using the AUC of the receiver operating character (ROC) curves. Then, the concordance between the predicted and the nomogram for FL/DLBCL actual survival probability was shown using a calibration plot.

### 2.5. Statistical Analysis

To measure survival, Kaplan–Meier survival curves were plotted. Then, the hazard ratios (HR), 95 percent confidence intervals for death, and *P* values for each clinicopathological parameter were calculated with the log-rank test. Clinicopathological factors that were significant in univariate analyses were identified using a two-sided test with a *P* < 0.05 threshold of significance. Then, those variables were used for the stepwise construction of multivariate Cox regression models, with *P* < 0.05 as a significance threshold. The nomogram was constructed on the grounds of the Cox model parameter estimates in the primary cohort. The time-dependent receiver operating characteristic (tROC) was used to compare with traditional prognostic models. The corresponding areas under curve (tAUC) were used to evaluate model discrimination. All statistical work was conducted with ggplot2, Hemic, rms, and the tROC package in R statistical software version 4.0.3 (http://www.R-project.org) (2020-10-10).

## 3. Results

### 3.1. The Characteristic and Outcome in Three Groups

The main baseline characteristics of the 121 FL/DLBCL patients are listed in Supporting Table 1. The median age of diagnosis was 57 years (range: 22–79 years). Seventy-six cases (64%) exhibited FL grade 1–3a, while 45 (36%) exhibited FL grade 3b at diagnosis. Seventy-one cases (59%) were of GCB origin, and 55 (41%) were of non-GCB origin. Four hundred seventy-one patients were diagnosed with pure FL 1–3a (grade 1, 67 cases; grade 2, 321 cases; and grade 3a, 83 cases) (Supplementary Table 2). Among 529 de novo DLBCL cases, 252 (48%) were of GCB origin, and 277 (52%) were non-GCB. Kaplan–Meier survival curves of three groups in our investigation are illustrated in Figures 1(a) and 1(b). Pure FL 1–3a, FL/DLBCL, and *de novo* DLBCL groups showed a 5-year PFS of 70%, 59%, and 48% (*P* < 0.05). The 5-year OS values were 80%, 70%, and 60% (*P* < 0.05) for pure FL 1–3a, FL/DLBCL, and *de novo* DLBCL groups, respectively. Figures 1(c) and 1(d) show three groups receiving treatment with R-chemotherapy regimens. The PFS and OS of FL/DLBCL compared with pure FL 1–3a and *de novo* DLBCL groups with a 5-year PFS were 75%, 66%, and 56% (*P* < 0.05) and a 5-year OS of 88%, 76%, and 65% (*P* < 0.05), respectively.

### 3.2. The Outcome of FL/DLBCL Subtype Groups

According to the proportion of the DLBCL component, the outcomes of the 121 FL/DLBCL patients were analyzed. Differences in terms of both PFS and OS were not significant (Figures S1a and S1b). In addition, PFS and OS curves according to FL grade are presented in Figures S1c and S1d. These show that FL 1–3a/DLBCL patients demonstrated a significantly better outcome than FL 3b/DLBCL (*P* < 0.01) patients. Finally, COO subtype analysis show that non-GCB FL/DLBCL patients demonstrated a significantly worse prognosis than GCB FL/DLBCL patients (*P* < 0.01) (Figures S1e and S1f).

### 3.3. Univariate and Multivariate Analysis for OS

To identify the clinical prognostic factors for FL/DLBCL patients, we performed univariate analysis, which was related to poor OS. Significant correlations between presence of B-symptoms upon diagnosis, such as ECOG ≥ 2, Ann Arbor stage III–IV, lymph node area involvement ≥ 2 upon diagnosis, FL grade of 3b, COO non-GCB, extranodal involvement, elevated serum LDH, serum *β*2m, and rituximab-containing regimens, are summarized in Table 1. Cox's multivariate proportional hazard analyses were carried out after including all statistically significant clinicopathological parameters. These include FL grade 3b (HR 15.393, 95% CI 4.575, 51.788, *P* < 0.001), Ann Arbor stage III–IV (HR 3.881, 95% CI 1.080, 13.945, *P* = 0.038), and COO non-GCB (HR 4.236, 95% CI 1.238, 14.490, *P* = 0.021) and were independently prognostic for worse OS (Table 1).

### 3.4. Prognostic Index Construction and Internal Validation

Based on the findings of Cox's multivariate proportional hazard analysis, we proposed a nomogram for the prediction of 3- and 5-year OS. FL grade, Ann Arbor stage, and COO were incorporated into the nomogram (Figure 2). Next, we added the points for each patient and then divided these 121 FL/DLBCL patients by a quartile into four risk groups according to each patient's total points (Supplementary Table 4). CPPI showed a predicted 3-year OS of 97%, 74%, 57%, and 13% (*P* < 0.01) and 5-year OS of 94%, 66%, 42%, and 0% (*P* < 0.01) (Figure 3(a)). The predictive accuracy for 3- and 5-year OS as estimated using the AUC was 0.780 (95% CI, 0.691–0.873) and 0.870 (95% CI, 0.791–0.959), respectively. This is superior to that of the IPI, FLIPI, and FLIPI2 (ranging from 0.540 to 0.721, *P* < 0.01) (Figures 4(a) and 4(b)). The calibration plot for the likelihood of 3- and 5-year OS revealed a strong relationship between the nomogram's forecast and the observed outcome (Figures 4(c) and 4(d)). The predictive capacity with risk stratifications of the CPPI was more favorable in FL/DLBCL patients.

All 121 patients with FL/DLBCL were assigned at random to the internal validation cohort A (*n* = 72) or the internal validation cohort B (*n* = 49). Kaplan–Meier survival curves identified four risk groups accurately in both internal validation cohorts (Figures 5(a) and 6(a)). As measured by the AUC, the predictive accuracy of CPPI for 3- and 5-year OS was 0.779 (95% CI, 0.653–0.906) and 0.860 (95% CI, 0.744–0.976) in the internal validation cohort A (Figures S2a and S3a). According to the measurement of AUC, 3- and 5-year OS was 0.791 (95% CI, 0.656–0.926) and 0.906 (95% CI, 0.809–1.004) in the internal validation cohort B (Figures S2b and S3b). The calibration plot for the likelihood of 3- and 5-year OS revealed a strong relationship between the nomogram's forecast and the actual observed outcome (Figures S2c, S2d, S3c, and S3d).

### 3.5. Comparison with Traditional Prognostic Models

In patients with FL/DLBCL, Kaplan–Meier survival curves were plotted to estimate survival in the primary cohort and internal validation cohorts A and B. The predictive power of the CPPI with specified risk stratifications was better in FL/DLBCL patients (Figures 3(a), 5(a), and 6(a)). Additionally, the IPI was unsatisfactory for discriminating between any of the low-intermediate risk, high-intermediate risk, and high-risk groups (Figures 3(b), 5(b), and 6(b)). Furthermore, the FLIPI and FLIPI2 were unsatisfactory for stratifying between any intermediate-risk and high-risk groups in the study (Figures 3(c), 5(c), 6(c), 3(d), 5(d), and 6(d)).

In internal validation cohorts A and B, the CPPI outperformed IPI, FLIPI, and FLIPI2 in terms of accuracy levels. The AUCs of the CPPI in the internal validation cohorts A and B of 3-year OS (0.779; 95% CI, 0.653–0.906 and 0.791; 95% CI, 0.656–0.926, respectively) were high in comparison to those of the IPI, FLIPI, and FLIPI2 (*P* < 0.01) (Figures S2a and S2b). The AUCs of the CPPI in the internal validation cohorts A and B of 5-year OS (0.860; 95% CI, 0.744–0.976 and 0.906; 95% CI, 0.809–1.004, respectively) were high in relation to those of the IPI, FLIPI, and FLIPI2 (*P* < 0.01) (Figures S3a and S3b). The computed positions for the 3- and 5-year OS calibration plots were close to the diagonal line. The CPPI displayed better levels of accuracy for predicting survival in our study. These results indicate that the nomogram was an accurate and useful tool for the prediction of OS in patients with FL/DLBCL.

## 4. Discussion

Upon initial diagnosis, about 13% of individuals with newly diagnosed DLBCL demonstrated a concomitant indolent NHL, 8% demonstrated FL, and 5% demonstrated other indolent NHLs [6]. FL/DLBCL is referred as “transformed lymphoma upon diagnosis” or “early transformation.” In contrast, some researches consider FL/DLBCL as “composite lymphoma” [20, 34, 35]. We included all patients consecutively diagnosed with FL/DLBCL, pure FL 1-3a, or *de novo* DLBCL in our single center. After histology review, 1,121 cases of patients corresponded to these criteria. All patients received treatment of combined chemotherapy with or without rituximab. The outcomes of FL and DLBCL showed significant improvements in the past decade, using monoclonal anti-CD20 antibody rituximab combined immunochemotherapy as the standard therapy. However, in this retrospective study, fifty (41%) patients did not receive rituximab-containing regimens. Survival analysis confirmed that FL/DLBCL patients demonstrated intermediate survival between pure FL 1-3a and *de novo* DLBCL. Based on the findings of our study, patients with FL/DLBCL at diagnosis represent a lymphoma group distinct from pure FL 1–3a and *de novo* DLBCL groups. Few studies addressed this issue previously. Therefore, further discussing the risk factors that impact the poor prognoses and comparing the prediction capacity of traditional prognostic models are imperative, including IPI, FLIPI, and FLIPI2, in FL/DLBCL patients.

The new World Health Organization (WHO) classification of lymphoma suggests further subdivision of FL3 into grades 3a and 3b so that the proportion of involvement by DLBCL should also be reported. In our study, the proportion of the DLBCL component cannot predict for PFS and OS. However, the clinical implications of these features remain controversial. In the prerituximab era, most studies suggest that the proportion of DLBCL component predicted for EFS but not OS. Interestingly, in the rituximab era, the widespread use of rituximab-based chemoimmunotherapy significantly extended the survival in all risk groups. However, no significant differences were found in terms of either PFS or OS in the initial characteristics, according to the proportion of DLBCL component. It is accepted that FL grading (1–3) offers a degree of prognostic utility [1, 36]. Many FL 3b patients exhibit disease and treatment outcomes more like those of aggressive lymphoma patients despite exhibiting intact follicular architecture [18]. In contrast to FL 1–3a, the FL 3b relapse rate in some series is higher [37, 38]. However, the impact of histological grading on prognosis in FL/DLBCL patients remains unclear. Our results suggest that FL 3b/DLBCL patients may demonstrate a worse prognosis than FL 1-3a/DLBCL patients, similar to the results of previous studies [19]. Importantly, the multivariate analysis further confirmed that FL 3b/DLBCL could be used as a prognostic factor for FL/DLBCL.

Previous studies confirmed that COO assignments are valuable in predicting patient outcomes and immunochemotherapy responses in DLBCL [39, 40]. To our knowledge, limited data exists describing the COO in FL/DLBCL patients. In our study, seventy-one patients (59%) were of GCB phenotype, and fifty patients (41%) were of the non-GCB subtype. These figures differed from previous studies [6, 19], but they were supported by others [18]. Interestingly, COO offered prognostic value in individuals with FL/DLBCL, demonstrating that patients with non-GCB-type FL/DLBCL most often exhibited a reduced OS relative to those with GCB-type disease. Although, rituximab was associated with improved survival outcomes in both disease types. These results are relevant given that they indicate the potential for tailoring treatments based upon underlying COO subtype to overcome negative outcomes in those with non-GCB type disease.

The nomogram is a mathematical model based on a visual expression that combines biological, clinical, and pathological variables to determine the likelihood of a clinical occurrence [41, 42]. It has been manifested from investigations focused on a variety of malignancies for which nomograms allow superior predictive accuracy for clinical results in comparison to the previously used predictive systems [43, 44]. Accordingly, we developed the CPPI based on nomogram, an OS predictor index based on clinical and pathological routine characteristics that accurately stratify FL/DLBCL patients into four risk groups. The CPPI integrates FL grade, COO, and Ann Arbor stage as the new OS predictor index. The nomogram based on a single institutional patient cohort has been internally verified to predict survival in FL/DLBCL patients. Also, CPPI assesses individual FL/DLBCL patients' risk. The results show that the nomogram accurately predicts OS. Notably, all these prognostic factors are easily available during diagnosis. The nomogram's clinical variables may be recorded by any doctor communicating with patients presenting with FL/DLBCL, thereby increasing its usefulness. Further, the internal validation confirmed that the CPPI is a robust risk stratification tool for FL/DLBCL.

Several traditional models, including the IPI, FLIPI, and FLIPI2, have been validated in DLBCL and FL patients [22, 45]. In FL/DLBCL, however, the capacity to predict survival and risk identification of this traditional model were decreased. Since its origin relates to the clinical and pathological attributes that are easily attainable at diagnosis, CPPI is a viable option. Unlike other prognostic systems, CPPI demonstrates an improved capacity to stratify patients into distinct risk categories and an improved ability to predict OS. In FL/DLBCL patients, the CPPI's AUC for OS prediction was far more accurate than that of the IPI, FLIPI, and FLIPI2. As far as we are aware, this is unprecedented work focused on constructing a FL/DLBCL prognosis nomogram using the clinicopathological parameters of patients, as well as the first one designed based on an FL/DLBCL database in the Chinese population.

This study sought to gauge the odds of 3- and 5-year OS through the utilization of multivariate Cox proportional hazard models including FL grade, COO, and Ann Arbor stage as a novel independent OS predictor in FL/DLBCL patients. From a single institutional patient population, the CPPI has been generated and internally validated as being dependable as an instrument for survival prediction in those with FL/DLBCL. Additionally, CPPI provides the risk assessment for each FL/DLBCL patient. The results show that it demonstrates a high degree of accuracy in predicting OS. Furthermore, all these variables are readily assessed at diagnosis. The clinicians caring for patients with FL/DLBCL will be able to document the clinical variables included in the nomogram, thus enhancing its practical utility.

Although the CPPI exhibited higher levels of accuracy in predicting OS, our prognostic index exhibits significant limitations. First, this retrospective study design used a small patient cohort generated from a single center. Our conclusions, however, could be prospectively verified in normal patient care and used to guide treatment plans. Second, the research was conducted using a database of clinicopathological characteristics. As a result, if this nomogram could be used with individuals from nonendemic locations and different geographical regions is uncertain.

## 5. Conclusion

The CPPI demonstrates superior prognostic ability compared to the IPI, FLIPI, or FLIPI2 in FL/DLBCL patients. Its basis on FL grade, COO, and Ann Arbor stage promises to be a simple, accessible, and effective tool for identifying high-risk patients. It would be useful in routine clinical practice, allowing treatment approaches to be modulated accordingly. However, these prognostic models require further validation in prospective analyses to confirm their clinical relevance.

## Figures and Tables

**Figure 1:** Kaplan–Meier survival curves of the pure FL 1–3a, FL/DLBCL, and *de novo* DLBCL groups (a, b) and treatment with R-chemotherapy regimens (c, d).

**Figure 2:** Nomogram for patients with FL/DLBCL. To utilize the nomogram, the patient's value is placed on each variable axis, and a line is drawn upwards to calculate the number of points awarded for each variable value. On the total point axis, the sum of these numbers is shown, and a line is drawn downwards to the survival axis to calculate the 3-year and 5-year OS probabilities.

**Figure 3:** Kaplan–Meier survival curves of the CPPI (a), IPI (b), FLIPI (c), and FLIPI2 (d) in the primary cohort of FL/DLBCL. Abbreviations: IPI: International Prognostic Index; FLIPI: Follicular Lymphoma International Prognostic Index; FLIPI2: Follicular Lymphoma International Prognostic Index 2; LR: low risk; LIR: low-intermediate risk; HIR: high-intermediate risk; HR: high risk.

**Figure 4:** ROC curves for predictions of 3- and 5-year OS in different models (a, b) and calibration curves (c, d) in the primary cohort. Abbreviations: ROC: receiver operator characteristic; AUC: area under the curve.

**Figure 5:** Kaplan–Meier survival curves of the CPPI (a), IPI (b), FLIPI (c), and FLIPI2 d) in internal validation cohort A. Abbreviations: IPI: International Prognostic Index; FLIPI: Follicular Lymphoma International Prognostic Index; FLIPI2: Follicular Lymphoma International Prognostic Index 2; LR: low risk; LIR: low-intermediate risk; HIR: high-intermediate risk; HR: high risk.

**Figure 6:** Kaplan–Meier survival curves of the CPPI (a), IPI (b), FLIPI (c), and FLIPI2 (d) in internal validation cohort B. Abbreviations: LR: low risk; LIR: low-intermediate risk; HIR: high-intermediate risk; HR: high risk.

**Table 1:** Univariate and multivariate analysis of prognostic factors for OS in FL/DLBCL groups.

Parameter	Univariate analysis			Multivariate analysis		
	HR	95% CI	*P*	HR	95% CI	*P*
Age ≥ 60 years	1.177	[0.567, 2.441]	0.662			
DLBCL component ≥ 50%	0.651	[0.296, 1.431]	0.285			
FL grade 3b	16.845	[5.830, 48.671]	<0.001	15.393	[4.575, 51.788]	<0.001
Cell of origin non-GCB	7.033	[2.856, 17.318]	<0.001	4.236	[1.238, 14.490]	0.021
Ann Arbor stage III–IV	10.661	[3.689, 30.807]	<0.001	3.881	[1.080, 13.945]	0.038
Bone marrow involvement	8.640	[3.504, 21.306]	0.106			
ECOG ≥ 2	3.820	[1.802, 8.096]	<0.001			
B-symptoms present	2.327	[1.115, 4.858]	0.025			
Number of nodal areas ≥ 2	2.154	[1.028, 4.513]	0.042			
Extranodal involvement	2.287	[1.011, 5.175]	0.047			
Splenic involvement	0.576	[0.234, 1.416]	0.229			
Hemoglobin < 12 g/l	0.784	[0.273, 2.256]	0.652			
Serum LDH elevated	2.902	[1.348, 6.248]	0.006			
Serum *β*2m elevated	2.302	[1.097, 4.831]	0.027			
Rituximab-containing regimens	3.039	[1.409, 6.552]	0.005			

Abbreviations: DLBCL component: FL with the percentage of DLBC component; non-GCB: nongerminal center B-cell like DLBCL; ECOG: Eastern Cooperative Oncology Group; LDH: lactate dehydrogenase; *β*2m: *β*2-microglobulin; CI: confidence interval; HR: hazard ratio.

## Data Availability

The data that support the findings of this study are available from the corresponding author upon reasonable request.

## Supplementary Materials

Supplementary Materials Supplementary Table 1: the baseline characteristics of FL/DLBCL groups. Supplementary Table 2: the baseline characteristics of pure FL 1-3a groups. Supplementary Table 3: the baseline characteristics of de novo DLBCL groups. Supplementary Table 4: prognostic score from nomogram. Supplementary figure 1: Kaplan-Meier survival curves according to proportion of DLBCL component (a, b), FL grade (c, d), and cell of origin (e, f). Abbreviations: DLBCL component: FL with the percentage of DLBC component; GCB: germinal center B-cell like DLBCL; non-GCB: nongerminal center B-cell like DLBCL. Supplementary figure 2: ROC curves and calibration curves for predictions of 3-year OS in internal validation cohort A (a, c) and internal validation cohort B (b, d). Abbreviations: ROC: receiver operator characteristic; AUC: area under the curve. Supplementary figure 3: ROC curves and calibration curves for predictions of 5-year OS in internal validation cohort A (a, c) and internal validation cohort B (b, d). Abbreviations: ROC: receiver operator characteristic; AUC: area under the curve.
